# A Deep Learning Method for Intelligent Analysis of Sports Training Postures

**DOI:** 10.1155/2022/2442606

**Published:** 2022-07-31

**Authors:** Yuqin Sun, Youliang Li

**Affiliations:** ^1^Jiangxi Environmental Engineering Vocational College, Ganzhou 341000, China; ^2^Institute of Physical Culture, East China University of Technology, Nanchang 330013, China

## Abstract

With the further research of artificial intelligence technology, motion recognition technology is widely used in posture analysis of sports training. However, the interference of light, Angle, and distance in real life makes the existing model unable to focus on the expression of human movements. Aiming at the above problems, this paper proposes a motion training attitude analysis method based on a multiscale spatiotemporal graph convolution network. Firstly, the spatiotemporal image of the skeleton is constructed, and then the convolution operation is performed on the spatiotemporal image of the skeleton. Finally, the convolution results are linearly weighted and fused to capture the characteristics of action types with different time lengths. At the same time, the algorithm increases the processing of some important information loss and increases the randomness of the data set. Experimental results show that the proposed algorithm can adapt to the behavior changes of different complexity, and the model performance and recognition accuracy are significantly improved.

## 1. Introduction

With the rapid development of artificial intelligence, image pattern recognition technology has played an essential role in People's Daily life in recent years [1]. Human motion recognition models spatiotemporal information based on presegmented temporal sequence [2]. Learn the semantic and motion characteristic information contained in the video to build the mapping between the video content and action categories so as to classify human behavior. Motion recognition is widely used in video understanding, intelligent monitoring, pedestrian tracking, human-computer interaction, and other fields [3].

In each attempt of the same movement, the joint trajectories of the corresponding joints generally have similar basic shapes [4]. However, due to the influence of various factors, the trajectory of the joint of the same person will also have certain changes, which will affect the correct recognition of the movement [5]. These factors can be generalized into space and time. The spatial factors mainly include the change of shooting Angle leads to the change of coordinate system to describe the action. Body shape and size of different participants lead to changes in skeleton scale, and the motion amplitude of different participants leads to differences in trajectory scale [6]. The time factor represents scale scaling along the time dimension. Different participants perform the same action, or the same person repeats the action at different speeds [7]. The spatial factors are modeled as affine transformation in 3-dimensional space to deal with these differences and changes. The scale transformation of time dimension is relatively complex, and it is generally simplified linearly into uniform time scale scaling, which is modeled as affine transformation in a 1-dimensional space of time dimension [8]. The combination of these two affine transformations is the space-time biaffine transformation.

Human motion estimation should simultaneously consider the detection and connection of multiple human key points. Literature [9] proposed that a convolution pose machine generates the initial pose and then applies integer linear programming to obtain the final pose. Literature [10] adopted human body detection based on FAST-CNN. Literature [11] proposed an attitude partitioning network for node detection and intensive regression. The OpenPose model proposed in the literature [12] uses a method called partial affinity field, which can encode the position and direction of limbs and correctly connect key points in this way. Graph Convolutional Network (GCN) can effectively extract non-European data features. Literature [13] firstly applies Graph Convolutional network to bone-based action recognition and proposes the spatial-temporal Graph Convolutional Networks (ST-GCN) model. Literature [14] designed a dual-flow adaptive graph convolutional network based on ST-GCN and introduced a nonlocal block adaptive method to learn the connections between nodes. In order to obtain richer joint correlation dependencies, a motion structure graph convolution network (AS-GCN) was proposed in the literature [15]. Literature [16] proposed motif-based graph convolution to encode hierarchical spatial structure and used variable time-intensive blocks to mine information facing different time ranges in human bone sequences.

Therefore, the key to behavior recognition lies in designing a network model to extract dynamic information from the human skeleton [17]. Inspired by the study of graph convolution (GCN), a motion training attitude analysis method for a multiscale spatiotemporal graph convolution network is proposed in this paper. Considering the spatial structure of preserving the natural connection of joints in motion in bone information, the skeleton as a whole is input to graph convolution network as a topology. Combined with multiscale TCN, the time dynamic modeling of bone can integrate the bone information from the spatiotemporal dimension to learn more effective information to improve the model effect of behavior recognition.

The innovations and contributions of this paper are listed below.

1. Construct the bone space-time map and conduct convolution operation on the bone space map;
2. Weighted fusion of skeletal convolution was performed to capture the characteristics of motion types with different time lengths;
3. Multiscale convolution is carried out at the base of each volume to obtain features at different scales.

This paper consists of four main parts: the first part is the introduction, the second part is the methodology, the third part is the result analysis and discussion, and the fourth part is the conclusion.

## 2. Methodology

### 2.1. Skeleton Action Recognition Based on Graph Convolution

Graph representation is the primary problem of skeleton action recognition. It is very important to increase the flexibility of the network and improve the efficiency of information transfer between nodes while preserving the original connection relationship of bones.

#### 2.1.1. Diagram

The coordinates of human key points can be obtained by using sensors to obtain position information or attitude estimation of behavior video, denoted as *q*_*x*_=(*i*_*x*_, *j*_*x*_, *k*_*x*_). A simple skeleton diagram can be represented based on the natural adjacency between key points, denoted as *A*_*x*_=(*Q*_*x*_; *G*), where *Q*_*x*_ represents the key point set of frame *x*. *G* is the adjacency matrix, size *T∗T*. *T* is the number of key points. The adjacency matrix contains only 0 and 1 values, where (*x*, *y*)=1 indicates that there is a directly connected edge between the *i*th key point and the *j*th key point. (*x*, *y*)=0 means there is no directly connected edge between the *i*th key point and the *j*th key point. Therefore, the complete video skeleton sequence can be represented as a stack of bones for each frame, i.e., *A*=(*A*_1_; *A*_2_; …; *A*_*x*_).

#### 2.1.2. Application

Skeleton sequences are usually represented as *C* × *N* × *T* matrices as the original inputs of the network. *C* indicates the number of channels. *N* is the number of frames. *T* indicates the number of key points. The existing methods mostly deal with skeleton sequences in spatial and temporal dimensions.

In spatial domain, ACT is used to extract features. Based on the representation method of the bone graph in Section 2.1.1, the information of neighbor nodes is aggregated, as shown in the formula .

(1) $$\begin{array}{c} f_{\text{out}}=\sum_{z}^{Z_{z}}M_{z}\left(f_{\text{in}}G_{z}\right)⊗W_{z}, \end{array}$$

where *W*_*z*_ is A learnable parameter. ⊗ is the product of elements between two matrices. *Z*_*q*_ is the number of subsets of the adjacency matrix. *M*_*z*_ is a learnable parameter with the size of *C*_out_ × *C*_in_ × 1 × 1, which is used to adjust the channels of the feature graph. *G*_*z*_ is the subset of adjacency matrix obtained according to the subgraph partitioning strategy.

(2) $$\begin{array}{c} G_{t}=\Lambda^{-1/2}\left(\bar{G}+X\right)\Lambda^{-1/2}, \end{array}$$

where $\bar{G}$ is the adjacency matrix. *X* is the identity matrix. *G* is the degree matrix, $\Lambda^{xy}=\sum_{y}\left(\overset{⟶}{G^{xy}}+X^{xy}\right)$. *G*_*t*_ is the normalized adjacency matrix.

In the time domain, the existing methods mostly adopt one-dimensional convolution to fuse the features of the same key point in different frames.

### 2.2. Convolution of Space-Time Maps Based on Bones

#### 2.2.1. Skeleton Space-Time Map Construction

The skeleton of the human body is also a collection of points and edges made up of joints and limb connections, conforming to the definition of the graph. Therefore, graph convolution can be used for the human skeleton. However, a problem that needs to be considered is that it is not a piece of static information but a series of data with continuous time series in human movement. To make better use of graph convolution to extract dynamic information of bone, in addition to the spatial edges of natural connection of bone nodes in space, time edge information between different time frames is added to describe the change characteristics of behavior in time series. The traditional graph convolution is extended to the time neighborhood, as shown in Figure 1.

The structure *A*(*Q*, *E*) of the space-time skeleton diagram is formed by the connection between the nodes of the graph and the space-time edges. The information in the graph includes *T*, the number of key nodes, and *N*, the number of frames in an input video. *Q*_*x*_ represents the eigenmatrix corresponding to each node. Therefore, the feature matrix set of all nodes in the t-frame can be obtained as shown in the formula:

(3) $$\begin{array}{c} Q=\left\{q_{nx}|n=1,\ldots ,N,x=1,\ldots T\right\}, \end{array}$$

where the feature vector of the *xth* node in a single frame is represented by *f*(*q*_*x*_). It contains the coordinates and confidence of each joint. There are two main steps in the construction of a bone space-time map. The first step is to obtain the original connection of the human skeleton in the movement process without the need for manual design. The human body node information in the video sequence can be obtained through an openpose tool or related equipment, and the natural body bone structure can be constructed based on the obtained node information. The second step is to connect the same joint between adjacent frames on the basis of the spatial map to form the space-time map of the skeleton sequence. Multiple frames of the continuous skeleton also need to be connected to the time edge. Therefore, the set of edges consists of two parts, represented by *E*_*s*_ and *E*_*f*_ respectively, as shown in the following formula:

(4) $$\begin{array}{c} E_{s}=\left\{q_{x}q_{ly}|\left(x,y\right)\in B\right\},\\ E_{f}=\left\{q_{xx}q_{\left(n+1\right)x}\right\}, \end{array}$$

where *E*_*s*_ is the connection of bone points within a single frame. *E*_*f*_ is the connection between different frames of the same bone point. The trajectory information of the human movement process with time is described by constructing a space-time diagram.

#### 2.2.2. Convolution of Skeletal Space Map

First, the spatial information of the skeleton is modeled. According to the definition of graph convolution, the formula of the convolution network can be extended. Take convolution operation as an example, as shown in the formula

(5) $$\begin{array}{c} f_{\text{out}}\left(I\right)=\sum_{b=1}^{Z}\sum_{m=1}^{Z}f_{xt}\left(u\left(i,b,m\right)\right)\cdot m\left(b,m\right). \end{array}$$

There are two main functions, sampling function and weight function, respectively. The sampling function *u* is mainly used to obtain pixels in the neighborhood of *i*. A grid-like region of size *Z∗Z* around the center point *i*. The weight matrix *m* indexes the data in the grid region selected by the sampling function *u* in a certain spatial order. The weight relation between each neighborhood pixel and the center point can be obtained by inner product operation between the weight matrix *m* and the sampling region. This formula can be modified to apply to the bone space-time map, and the sampling function and weight function can be improved, respectively. In the previous section, the space-time skeleton diagram was constructed to obtain the set *Q* of nodes. So the center of the sampling function becomes the skeleton node *q*. The sampling region becomes a collection of nodes neighboring nodes and is represented by *H*(*q*_*nx*_)={*q*_nyn_*|d*(*q*_*ny*_, *Q*_*nx*_ > =*Z*)}, where *d* represents the minimum distance from the sampling point *q*_*n*_. *Z* stands for the set with distance range *Z*. Here, the value of *Z* is 1 to select the neighborhood set whose distance node is 1.

Then the weight function is redefined. Since graph convolution has no fixed order in space, it is necessary to divide the neighborhood set *H*(*q*_*n*_). Assuming the number of subsets divided is A label mapping function encodes *T*, each of them. (*q*_*x*_)=*H*(*q*_*x*_)⟶{0,1,…*T*}So that the points in the neighborhood are mapped to specific subsets after partition so that they have the same label, and a new weight function can be obtained. The details are expressed in the formula

(6) $$\begin{array}{c} m\left(q_{nx},q_{ny}\right)=m^{\prime }\left(l_{nx}\left(q_{ny}\right)\right). \end{array}$$

Therefore, by extending formula (6) and applying the new weight and sampling function, the graph convolution expression of bone can be obtained as shown in the formula

(7) $$\begin{array}{c} f_{\text{out}}\left(q_{xn}\right)=\sum_{q_{ny}\in H\left(q_{nxn}\right)}\frac{1}{K_{xx}\left(q_{ny}\right)}f_{xt}\left(u\left(q_{nx},q_{ny}\right)\right)\cdot m\left(q_{xy},q_{xy}\right). \end{array}$$

Among them, *K*_*nx*_(*q*_*ny*_)=|{*q*_*nz*_*|l*_*nx*_(*q*_*nz*_)=*l*_*nx*_(*q*_*nx*_)}| is equal to a subset of the base and is used to reduce the influence of different subsets of the output.

#### 2.2.3. Multiscale Time Convolution

Different behavior types have different time characteristics. The duration of the action also varies depending on the type of action. A multiscale method is proposed to convolve action types with different periods to describe the characteristics of action variation better. Then, the convolution results are linearly weighted and fused so that the network model can simultaneously capture the characteristics of action types of different time lengths and adapt to the behavior changes of different complexity.

The formula of graph convolution is extended to time domain modeling. The node neighborhood analyzed in the previous section is the bone graph connection within a single frame. Next, the connection between the same nodes between its consecutive frames is considered, as shown in the formula

(8) $$\begin{array}{c} S\left(q_{xd}\right)=\left\{q_{ey}\left|d\left(q_{nx},q_{xy}\right)\leq Z,\right|v-n|\leq \left|\frac{\Gamma }{2}\right|\right\}, \end{array}$$

where Γ represents the span of the time axis. Its value determines the size of the convolution kernel at the time of convolution. In order to enable node *q*_*x*_ to generate corresponding neighborhood space in time and space dimensions, the tag mapping function constructed above needs to be modified as shown in the formula

(9) $$\begin{array}{c} l_{SN}\left(q_{qy}\right)=l_{nx}\left(q_{ny}\right)+\left(v-n+\left|\frac{\Gamma }{2}\right|\right)\times Z. \end{array}$$

#### 2.2.4. Framework Description of Multiscale Time Convolution Method

The single convolution kernel scale of traditional TCN is extended. Multiscale TCN (hereinafter referred to as mS-TCN) was adopted, and a convolution kernel with a time span of 2 *γ* was added to extract the behavior features with long duration, as shown in Figure 2. In the process of time convolution, a new convolution with a scale twice the size of the original convolution kernel is added to convolve time features, and the total number of convolution kernels remains unchanged. At this time, the network contains two convolution checks with different time spans for feature extraction of bone vectors. In this way, multiscale convolution can be carried out at each convolution layer to obtain the characteristics of the input bone information at different scales. Finally, the information extracted from the two convolution kernels is fused and input to SoftMax through average pooling to complete behavior classification. Its principle structure is shown in Figure 2.

The calculation process of each convolution kernel contained in multiscale time convolution is the same, and its principle is shown in the formula

(10) $$\begin{array}{c} f_{x}=f_{x-1}+M_{x}*\lambda f_{x-1}, \end{array}$$

where *f* is the output. *x* indicates the number of network layers. *M* represents the set of all filters at layer *x*. *λ* is Relu activation function. Let the number of original TCN network filters be *T*, then two convolution kernels with *T*/2 in number and *z∗*1 and 2*z∗*1 in size can be obtained through multiscale variation. The convolution operation is carried out on n-frame video, and the feature dimension of each node is *C*. Firstly, feature extraction of node *i*_*x*_ is carried out. Move along the direction of the time series according to step size 1. Move down after the completion of convolution to traverse all key nodes. In each convolution process, convolution results of two scales are connected to form convolution results, which are transferred and accumulated among the 10 network layers constructed in turn. Then, the final input of this network is the key node vector *I* after openpose processing. After multiscale convolution, *I* is convolved, respectively. The convolution process of the two spans is shown in the black solid line and dotted line box in the figure. Then, all the results after convolution are spliced, and the final result is linearly weighted fusion.

### 2.3. Application of Convolution of Multiscale Space-Time Graph

Space-time graph convolution is applied to behavior recognition. Firstly, the openpose processing tool will be used to estimate the posture of human behavior in the input video, and the marked joints of the human body will be connected to the skeletal output. Then, the coordinates of nodes of different frames are normalized by the BN layer. In this way, the influence of different dimensions can be eliminated, the influence of data characteristics on results due to different evaluation indexes can be reduced, and the comparability of data sets can be further enhanced. At the same time, the attention model layer is added to the whole network to learn the weights of adjacent nodes. Because the nodes are constantly changing during human movement, the modeling of each dynamic part has a different degree of relevance to the node connection. In running, for example, leg information is more important than neck information. Therefore, adding an attention layer allows the network model to autonomously learn the importance of each spatial edge. Then input graph convolution GCN and multiscale time convolution (MS-TCN) fusion network model. Finally, softmax classifier is used to complete the classification of human behavior. The overall network structure is shown in Figure 3.

#### 2.3.1. Data Preprocessing

Openpose can mark predefined key parts of the body such as the neck, shoulder, and arm. Then the marked joints are connected, that is, the extraction of the human skeleton. Here, the two people with the highest average confidence in each frame are selected, and the coordinate vectors of their key points are extracted as input.

Usually, each batch of video input into the network can be represented by a 5-dimensional matrix (*T*, *C*, *N*, *Q*, *W*), where *T* represents the number of videos in a batch. *C* is used to represent the features of the joint, that is, the coordinates of *i* and *j*, and the three features of confidence. *N* represents the number of key frames. *Q* is the number of joints. Since there are different numbers of nodes marked by openpose, the value of *Q* is different, so the final input network shape is (256, 3, 155, 20, 4).

#### 2.3.2. Subset Division

In the process of spatial graph convolution, it is necessary to divide the neighborhood of each node. Considering the characteristics of different behaviors and the spatial and temporal structure of nodes, the neighborhood is divided into three subgraphs according to the distance between the root node and the center of gravity (the average coordinate of all bone points). The sampling point serves as the root node of the selection. Take the distance *r*_*x*_ between the root node and the center of gravity as standard. If the distance between points in the neighborhood and the center of gravity *r*_*y*_ is greater than *r*_*x*_, it is divided into subset 1. If the distance from the center of gravity is less than *r*_*x*_, it is divided into another subset 2 as shown in the formula

(11) $$\begin{array}{c} l_{xy}\left(q_{xy}\right)=\left\{\begin{array}{cc} 0, & r_{y}=r_{x},\\ 1, & r_{y}<r_{x},\\ 2, & r_{y}>r_{x}. \end{array}\right. \end{array}$$

The divided subgraph has three subgraphs, as shown in Figure 4.

In this way, it can be divided into three subgraphs, representing centrifugal, centripetal, and stationary motion forms, respectively, which can more effectively capture the spatiotemporal information of behavior and action. The number of convolution kernels changes from 1 to 3, i.e., (1, 20, 20) to (3, 20, 20). Then according to the scale-invariant convolution property, the three convolution kernels are convolved, respectively. Then you take a weighted average (the same as the convolution), and you get the final result.

#### 2.3.3. Multiscale Time Convolution and Model Fusion

Another point that needs to be considered for the network is how to fuse the model effectively. The classifier adopted is softmax. All function outputs are mapped to (0, 1) outputs considering their function properties. To reflect the advantages of each model, linear weighted fusion is adopted, as shown in the formula

(12) $$\begin{array}{c} u_{\text{fusiona}}\left(j_{x}\right)=\alpha u_{g}\left(j_{x}\right)+\left(1-\alpha \right)u_{h}\left(j_{x}\right), \end{array}$$

where *α* is the parameter and *u* is the probability matrix. The behavior type output after model fusion can be obtained by operation according to the formula.

## 3. Result Analysis and Discussion

### 3.1. Experimental Settings

- Experimental platform. The graphics card is a single NVIDIA GeForce RTX2060 Super. The processor is Intel i5-10400F. The memory is 64 GB. The operating system is Ubuntu 19.10. The language is Python 3.8. CUDA version is 11.2, using PyTorch 1.6.0 framework.
- Related parameter settings. In order to make the size of the feature graph output by convolution of each layer graph match the size of the multichannel adaptive graph, the frame number of the skeleton sequence was uniformly set to 25 in the experiment. In order to compare the baseline method more fairly, other hyperparameter settings are consistent with the baseline method. Set the initial parameters of the network. See Table 1 for the entire network configuration.
- Data set setting. The dataset uses two recommended assessment settings, namely CS (cross subject) and SS(cross set number). To make the model more generalized, this paper adopts the same data setting approach as the baseline approach. The 3 d bones in each sequence were randomly rotated around the *X*, *Y,* and *Z* axes by a certain degree [−18°, +18°]. For data preprocessing, the data preprocessing method proposed in this paper is adopted.
- Training time. The model was trained using NTU-RGB + D120 data set on a single NVIDIA GeForce RTX2060 Super graphics card. The total training time of 120 epochs in each assessment setting was over 1.5 hours.

### 3.2. Universal Data Set Experiment

#### 3.2.1. Data Set

The NTU-RGB + D120 dataset is one of the most popular large-scale motion recognition datasets. The dataset contained 120 action categories, completed by 108 different subjects with 32 different settings, totaling 114 490 action samples. Of these, 538 samples were not available. The human skeleton in each action sample consists of 25 joints, each of which is represented by 3D coordinates. This dataset can be set in two ways. (a) Cross subject. The 108 subjects were divided into two groups, half for training and half for testing. The number of samples in the training set was 63 028, and the number of samples in the test set was 50 924. (b) Cross setup number. The 32 different set numbers were divided into two groups, with even numbers for training and odd numbers for testing. The number of samples in the training set was 54 468, and the number of samples in the test set was 59 484.

#### 3.2.2. Experimental Results and Analysis

In order to verify the effectiveness of the proposed algorithm on data preprocessing, different data preprocessing methods are used in experiments for both the proposed algorithm and the comparison model.

In order to make a fair comparison, bone sequence length was set to 25 in both data pretreatment methods. For data preprocessing, the data preprocessing method proposed in this paper is adopted. The experimental results in Figure 5 show that the recognition accuracy of the proposed algorithm is improved compared with other comparison algorithms when CS evaluation settings are used, with a maximum improvement of 5.95%. In the SS evaluation setting, the recognition accuracy of the proposed algorithm is also improved compared with other comparison algorithms, with a maximum improvement of 4.73%. The reason why the model recognition accuracy is improved is that the data preprocessing method proposed in this paper can effectively solve the problem of partial bone sequence frame loss caused by data preprocessing in other comparison algorithms. This avoids the loss of some important information and further increases the randomness of the data set. So the model can learn more important distinguishing features and increase the generalization of the model.

In order to verify the model performance under different values of parameter *α*, comparative experiments are carried out in this paper.  Table 2 shows the model performance of parameter *α* in the range of [0.2, 0.8]. The experimental results in Table 2 are verified, and the following conclusions are drawn: when *α* value is 0.6, the model has the best performance. Therefore, the value of *α* was set as 0.6 in subsequent experiments.

Experimental results of Table 3 show that single-scale time convolution will cause graph convolution in the model to degenerate into ordinary convolution. However, ordinary convolution cannot aggregate the features of correlative nodes, which leads to the degradation of model performance. Multiscale time convolution can effectively aggregate the features of correlative nodes and improve the model performance significantly. Compared with the single-scale time convolution model, the identification accuracy of the multiscale time convolution model is improved by 1.86% in the CS evaluation setting and 2.07% in the SS evaluation setting.

Figure 6 shows the comparison of convergence between the model in this paper and the comparative model. In order to make the comparison more fair, all models used the data preprocessing method in this paper. Compared with other models, due to the introduction of more information, the model in this paper can converge faster in the training process, and the convergence speed and degree are higher than other models.

As shown in Table 4, compared with reference [13, 18–20], reference [21] reduced the number of references by order of magnitude. Although the recognition accuracy was higher than the reference [13, 18, 19], it was lower than the reference [20]. Compared with the literature [21], the algorithm in this paper is not only lower in the number of parameters than the literature [21] but also significantly higher in recognition accuracy. Compared with other mainstream methods in Table 4, the method in this paper not only reduces the number of parameters by an order of magnitude, but also has higher recognition accuracy than other mainstream methods in Table 4. Experimental results show that the proposed method achieves a balance in recognition accuracy, computation amount and parameter number. Compared with other mainstream methods, it is more attractive and suitable for application scenarios with limited computing resources and requirements on recognition accuracy.

### 3.3. Exercise Training Data Set Experiment

This paper also constructs a real motion training pose video data set. The dataset was collected from 150 athlete videos and contained 2967 video clips. The main content is the movement training pose form six and the closing potential, subdivided into 20 kinds of movements.  Figure 7 shows an example of posture data set for sports training. In this paper, 2 000 video clips were used as training sets and 967 video clips as test sets. As listed in Table 5, most models can achieve good recognition effect in the taijiquan dataset.

The proposed method can achieve the performance listed in Table 5 for the following reasons:

1. The motion videos collected in this paper are all shot in front, and the subjects are always kept in the picture.
2. There is almost no extra object shielding the human body and background interference in the video scene. This results in high integrity and accuracy of extracted bone data, which is very important for motion recognition.
3. Subjects have a high degree of completion of performing video actions and fewer nonstandard actions. This allows the network to better extract features. Due to the addition of the causal coefficient as edge weight, this paper can highlight the main joints in the process of human movement, and its effect is still better than other methods. This shows that the graph convolution network based on joint causality is more biased towards some nodes.

## 4. Conclusion

Human motion recognition has been a research hotspot in the computer vision field in recent years. Posture analysis of sports training has a wide and potential application value in sports teaching, athlete training, and other fields. To better analyze the motion training posture, this paper proposes a motion training posture analysis method based on a multiscale spatiotemporal graph convolution network. To extract the features of motion information, the algorithm constructs a spatiotemporal graph convolution network from the construction level. Based on traditional image convolution, graph convolution is extended to describe better and capture the shape of motion. Experimental results show that the proposed algorithm can avoid the loss of some important information and further increase the randomness of the dataset. At the same time, the model performance under different values of parameter *α* is verified. The proposed method achieves a balance in recognition accuracy, computation amount, and parameter number, which is more attractive than other mainstream methods and more suitable for application scenarios with limited computing resources and requirements on recognition accuracy. In the future, more attention will be paid to action recognition with a smaller degree of differentiation. At the same time, we try to introduce adaptive methods to increase the research of limb orientation and length and analyze the motion training posture with feature fusion combined with the bone flow and node flow.

## Figures and Tables

**Figure 1:** Bone space-time map.

**Figure 2:** Multiscale time convolution network architecture.

**Figure 3:** The network structure.

**Figure 4:** Three subgraphs after partition.

**Figure 5:** Comparison of the effectiveness of pretreatment.

**Figure 6:** Comparison of convergence of different algorithms.

**Figure 7:** Schematic diagram of sports training posture dataset.

**Table 1:** Configure network model parameters.

Network parameters	The value
The layer number	10
Convolution time scale	16
Stride	1
Learning rate	0.001
Batch size	10
Epochs	150

**Table 2:** Comparison of model performance with different parameters *α*.

*α*	CS (%)	SS (%)
0.2	78.81	81.34
0.3	81.42	83.47
0.4	82.73	84.52
0.5	82.98	84.66
0.6	85.69	87.28
0.7	83.43	85.22
0.8	84.18	86.51

**Table 3:** Effectiveness comparison of multiscale time convolution.

Algorithm	CS (%)	SS (%)
Single-scale time convolution	84.61	86.18
Multiscale time convolution (proposed)	86.47	88.25

**Table 4:** Comparison of model parameters and recognition accuracy with other methods.

Algorithm	Param (M)	CS (%)	SS (%)
Literature [13]	3.11	70.71	73.24
Literature [18]	6.27	74.45	79.58
Literature [19]	6.98	77.78	78.93
Literature [20]	6.14	82.52	84.27
Literature [21]	0.73	81.17	82.74
Proposed	0.62	84.65	86.29

**Table 5:** Comparison of other technologies on sports training dataset (%).

Sports training dataset	Top-2	Top-6
Literature [13]	70.78	73.29
Literature [18]	74.41	79.54
Literature [19]	77.73	78.98
Literature [20]	82.56	84.24
Literature [21]	81.16	82.77
Proposed	84.68	86.32

## Data Availability

The labeled dataset used to support the findings of this study is available from the corresponding author upon request.
